This article has been retracted.

# Development of a Model System to Study Expression Profile of RAC2 Gene in Breast Cancer MDA-MB-231 Cell Line

**DOI:** 10.1155/2022/2077850

**Published:** 2022-03-24

**Authors:** Thogulva Sivakumar Harish, Polani Ramesh Babu, Anupama Shrestha, Balamuralikrishnan Balasubramanian, Arunachalam Chinnathambi, Sulaiman Ali Alharbi

**Affiliations:** ^1^Department of Genetic Engineering, Bharath Institute of Higher Education and Research, Selaiyur, Chennai-73, India; ^2^Center for Materials Engineering and Regenerative Medicine, Bharath Institute of Higher Education and Research, Selaiyur, Chennai-73, India; ^3^Department of Biotechnology, School of Science, Kathmandu University, P.O Box: 6250, Dhulikhel, Nepal; ^4^Department of Food Science and Biotechnology, Sejong University, Seoul, Republic of Korea; ^5^Department of Botany and Microbiology, College of Science, King Saud University, PO Box-2455, Riyadh 11451, Saudi Arabia

## Abstract

The RAC2 gene encoding GTPases involve cellular signaling of actin polymerization, cell migration, and formation of the phagocytic NADPH oxidase complex. Oncogenic mutations in the RAC2 gene have been identified in various cancers, and extensive research is in progress to delineate its signaling pathways and identify potential therapeutic targets in breast cancers. This paper explored developing a bioinformatics model system to understand the RAC2 gene expression pattern concerning estrogenic receptor status in breast cancers. We have used the MDA-MB-231 breast cancer cell line to identify RAC2 gene expression. To simplify the development of model system with one dataset, we retrieved the microarray dataset GSE27515 from the Gene Expression Omnibus (GEO) for the differential gene expression analysis. Then, network analysis, pathway enrichment analysis, volcano plot, ORA, and the up/downregulated genes were used to highlight genes involved in signaling network pathways. We observed that the RAC2 gene is upregulated in the GSM679722, GSM676923, and GSM679724 downregulated in the samples GSM676925, GSM676926, and GSM676927 from the GEO dataset. Our observation found that the RAC2 gene is upregulated in the estrogen receptor (ER) negative breast cancers and downregulated in ER-positive breast cancer, involving pathways such as focal adhesion, MAPK signaling, axon guidance, and VEGF signaling pathway.

## 1. Introduction

Breast tumors comprise phenotypically diverse populations of breast cancer cells, and in the current treatment modalities, the primary hormonal target is either ER protein or its receptor. In ER-positive breast cancer, ER is a therapeutic target, and ER-positive tumor includes lumina A and luminal B types [1–3]. Cancer stem cells (CSCs) initiate cancer development, which also mediates breast cancer metastasis and resistance to therapeutic drugs [4–13]. Solid tumor growth is generally enriched with CSCs that regulate growth and therapeutic relapse [14, 15]. CSCs are reported to regulate the intrinsic and extrinsic adaptation favoring their growth and survival [16]. In cancer research, a new term was “renewed” with the CSCs theory, whereby a subset of cells with stem cell-like properties are involved in cancer initiation.

Triple-negative breast cancer (TNBC) was characterized by its aggressiveness. However, by identifying suitable biomarkers and therapeutic targets, it is noticed that TNBC patients with reduced TNBC-specific therapeutic targets will not receive any benefits from the current treatment strategies [17, 18]. Therefore, valuable plans for using microarray and high-throughput sequencing technology are required to identify [19, 20]. Recently, bioinformatics methods have been widely used since it has the advantages of overcoming the inconsistency of data results of microarrays data and the limitation of the microvolume samples [21–23]. Using an integrated bioinformatics approach, a group of prostate cancer genes from GEO and TCGA databases with differentially expression screening was done with KEGG pathway analysis and protein-protein interaction networks were generated to predict core genes. This validated their results with RT-qPCR were analyzed and such studies resulted in the identification of critical genes and pathways from the microarray dataset [23–25]. In a few studies, gene expression patterns were used to classify the types of breast cancer based on molecular portrait [26, 27].

## 2. Materials and Methods

The Gene Expression Omnibus (GEO) is a helpful database in obtaining high-throughput functional gene expression data, which provides user-friendly methods for users to download and interpret data for functional genomics. This paper used GSE70690, GSE97342, GSE103019, GSE111122, and GSE27515 GEO datasets differential analysis in triple-negative breast cancer stem cells. Pathway enrichment analysis results in identifying omics genes, statistical analysis, visualization, and interpretation of the results [28]. The pathway topology uses additional information in databases like KEGG and PANTHER to complete gene-level statistics.

High-throughput omics technologies were used to show unbiased functional gene analysis and gene sets or network modules have been previously used to analyze molecular interactions [29–31]. In using Network Analyst, we were able to visualize and perform data analysis in the context of protein-protein interactions, which also provides details of uploaded functional gene dataset through over-representation and performs the pathway analysis for the datasets downloaded from the GEO database (GSE70690, GSE97342, GSE103019, GSE111122, and GSE27515). The PANTHER DB is used to find evolutionary relationships to analyze large-scale genomics and proteomics.

## 3. RNA Extraction and cDNA Synthesis

MDA-MB-231 (triple-negative breast cancer cell line) was obtained from NCCS, Pune, India, which was used to a culture in Leibovitz's Medium (Himedia, India), with 10% fetal bovine serum (FBS) in standard animal cell culture conditions using six healthy culture plates for 24 hrs. After incubation, 750 *μ*l of TRIzol was added to each well and repetitive pipetting lysed it. The lysed cells were used for RNA preparation and were quantified using Nanodrop, and cDNA was prepared stored at −20°C.

We used different bioinformatics tools to design a primer pair for PCR reactions. The original sequence in FASTA format was taken from the NCBI database. Then, the ORF of the series was found out using the ORF Finder tool, which can be accessed in NCBI itself. Further, the ORF from the respective sequence, primer BLAST, was performed to check the target specificity of the generated primer pairs. Later, the melting temperature and the annealing temperature of the generated primer pairs were analyzed from NEB's Tm Calculator tool. We were able to design the primer pairs for the respective RAC2 gene by the following steps. The gradient PCR was performed to standardize the PCR for the RAC2 gene. Plasmid DNA isolation is done using it as a vector and clones the gene RAC2. PcDNA 3.1+ is the plasmid that is used for this study. The pcDNA 3.1+ was inoculated in 6 ml of LB Broth and was cultured overnight.

## 4. Results and Discussion

The genes were retrieved from the microarray dataset from the genomic database by analyzing more than one dataset. To analyze the differential gene expression from the microarray data, we need to download two file formats: platform and series matrix files. The platform table is a tab-delimited table containing the information of the array definition. Platforms in GEO are submitted by the scientific community and represent various technologies, molecules types, and annotation conventions. The platform table also includes meaningful, trackable sequence identifiers such as GenBank/RefSeq accessions, locus tags, clone, clone IDs, oligo sequence, and chromosome locations. The series matrix file is a preprocess data file. In this study, though more datasets were available for analysis through GSE27515, due to development of a simple model system with one dataset to understand gene expression, we narrowed down our studies to one dataset, GSE27515. Further studies were given under consideration to extrapolate the further differential analysis using remaining dataset.

Once the series matrix and platform files are downloaded and uploaded to an online platform for comprehensive gene expression profiling and meta-analysis (Network Analysis), further, the dataset is subjected to quality check and normalization. Quality check is a process where the dataset's quality is analyzed, including correct sample size, experimental factors, and adequate gene annotations. There are three different plots used to view the quality check of the uploaded file. They are box plot, count sum, and density plot.

Normalization is a process of organizing data to minimize redundancy. Filtering increases statistical power by removing unresponsive genes before differential expression analysis (DEA). Proper normalization is essential to draw sound conclusions from the results of the DEA. The variance is a process, and the abundance filter is adjusted to change the number of genes excluded from the downstream analysis. The mean, standard deviation plot (MSD plot), and the principal component analysis plot (PCA plot) are the two plots that give us the information on the normalization of the dataset. The MSD plot provides information on the variation of the genes from a mean point. This will filter the unresponsive or represented in blue hexagons. The blue hexagons below the red lines depict the number of unresponsive genes.

The PCA plots can check the overall data quality and discover unusual patterns in the dataset. Samples can be plotted, making it possible to assess and verify the similarities and differences between models visually and determine whether samples can be grouped or not. The principal component analysis of the gene expression dataset GSE27515 in ER-negative and ER-positive breast cancer in the three-dimensional view is shown in Figure 1.

In Figure 1, each colored dot represents breast cancer samples plotted against its expression levels. The samples were colored according to their ER status; ER+ as red and ER− as blue. Using PCA plot, it was concluded that the estrogen receptor status was suggestive of having large influence on the gene expression profiles of the breast cancer cells. Hence, by subjecting the dataset to PCA, the PCA plots could provide potential insights about the choices of preprocessing and possible variable selections in dataset gene expression for further statistical analysis. PCA analysis clearly indicated that after normalization with respect to significant genes, ER-negative genes were absent as red color dot was not visible in the results, implying to investigate further in understanding detailed functional insignificance of such genes in breast cancer in ER-negative conditions. Volcano plot could be used to determine the number of upregulated and downregulated genes that were present in the given dataset (GSE27515). Hence, normalization was done so that we could easily separate the genes whose expression was altered in experimental conditions through the microarray analysis (Figure 2). Further, it could also separate the nonsignificant genes from significant genes from the expressed dataset.

In Figure 2, the blue-colored dots represent the number of the downregulated genes, and the red-colored dots represent the number of upregulated genes. The noncolored or grey colored dots represent the nonsignificant genes. According to the KEGG database, the highlighted genes are the genes involved in the pathways in cancer and focal adhesion (according to the KEGG database).

The volcano plot only allows the user to visualize the number of up- and downregulated genes present in the given dataset but also provides information on the expression patterns of individual genes.  Figure 3 shows the expression pattern of the RAC2 gene, and we can conclude the expression of RAC2 is upregulated in ER-negative breast cancer. The expression of RAC2 is downregulated in ER-positive breast cancer.

Heat-map is a standard method of displaying the gene expression data and visualizing it. Heat-map clustering is a method in which a group of samples is combined based on their gene expression pattern similarity. This method is proper when identifying the commonly regulated genes or biological signatures associated with a particular condition. There are two tools by which the heat-map clustering is done for the given dataset (GSE27515) (Figure 4).

The samples in the given dataset are combined, and the heat-map is constructed. In Figure 4, each row presents an individual sample. The gene expression levels are represented in blue shades and red shade boxes. The intensity of the colors ID is directly proportional to the unique gene expression level in that respective sample. If the intensity is more, then the expression is more, and if the intensity is faded, the expression is low. Upregulated genes are represented by red color, and downregulated genes are expressed by blue color. Here, the RAC2 gene is seen to be upregulated in the samples GSM679722, GSM676923, and GSM679724 and downregulated in the samples, GSM676925, GSM676926, and GSM676927. The KEGG database gives this heat-map. The over-representation analysis (ORA) is a comprehensive tool that uses various pathway databases for pathway enrichment analysis.

The ORA pathway enrichment analysis was done to the given dataset GSE27515. The blue arrow points at the RAC2 gene. From Figure 5, we can observe that the RAC2 gene is involved in many pathways, including focal adhesion, MAPK signaling, colorectal cancer, pathways in cancer, axon guidance, and VEGF signaling pathway. The pathway enrichment analysis was done using the KEGG database.

## 5. Functional Enrichment Analysis

The functional analysis of the dataset was done using the PANTHER tool.

The functional analysis of the dataset was done using the PANTHER tool.  Figure 6 shows the functional analysis of the biological process of the significant genes that were obtained from the dataset (GSE27515).  Figure 7 shows the pathway ontology of genes showing the presence of RAC2 playing role in cellular component organization in the biological process ontology of the dataset. Further investigation showed the involvement of RAC2 gene in various other biological processes like signal transduction.

The RAC2 was found to be in several functional pathways, including, RAS pathway, VEGF signaling pathways, integrin signaling pathway, and pathways in cancer and angiogenesis. The paths mentioned above are a part of the cAMP pathway and the RAC2 gene has a key role in them (Figure 8).

## 6. Analysis of Open Reading Frame from RAC2 mRNA

The open reading frame is a part of a sequence of different lengths. The FASTA format of the sequence is copy and paste in the given space in the ORF Finder tool. The minimum ORF length is set and the nested ORFs are removed. After submitting, we get the ORF length and its starting base pair and ending base pair along with the ORF sequence (Figure 9).

After determining the ORF for the sequence, primer pairs were designed based on common RAC gene amplification using Ras-related C3 botulinum toxin substrate 2 (rho family, GTP binding protein Rac2 sequences) (Figure 10). We considered the first twenty base pairs from the ORF sequence and used it as the forward primer sequence for our primer pairs. Then, we considered the last twenty base pairs as reverse primer sequence for our primer pairs. Then, the primer pairs checked for various physical parameters, GC content. Noncutting restriction enzymes were added before the primer pairs so that while going for digestion, our gene sequence would not be cut.

## 7. PCR Amplification of RAC2 Gene and cDNA Synthesis

Optimization of PCR conditions was done, the cDNA was synthesized, and cDNA was confirmed by performing PCR using the isolated RNA. The cDNA was successfully synthesized by adding the reverse transcriptase mix and performing the PCR under specific conditions.

In summary, we have retrieved the microarray dataset from the Gene Expression Omnibus for the differential gene expression. We have done the normalization and quality check of the microarray dataset of genes. Further, the list of significant genes was downloaded, which shows the list of upregulated and downregulated genes. Similar studies using cell lines were carried out to analyze expression data to identify drug targets. The MDA-MB-231 cell line has been used to study triple-negative breast cancers (TNBC), which is a mesenchymal type of stem cells and characterized by lack of estrogenic receptor (ER) and progesterone receptor (PR) and HER2 protein overexpression [17, 32]. Breast cancer cell line MCF7 and MDA-MB-231 were previously used to find a genetic marker and drug target by analyzing microarray GEO datasets [33]. In the current study, the network analysis and pathway enrichment analysis were done using GSEA as well as ORA and the up/downregulated genes were highlighted and narrowed down the novel upregulated gene RAC2 in triple-negative breast cancer cell line. We isolated RNA from the cultured MDA MD-231 cell lines and synthesized cDNA. The PCR conditions were optimized and amplified the RAC2 gene with 579 bp. Then, the plasmid DNA was isolated from *E. coli* harboring pcDNA3.1(+) human expression vector and confirmed by 1.5% agarose gel electrophoresis. In the current study, to simplify the RAC2 gene expression study, we considered 6 samples to develop the current model system, although in spite of dataset GSE27515 was available in GEO having more than six samples. Our studies determined a suitable model system to understand the therapeutic target identification through integrated bioinformatics approaches.

## Figures and Tables

**Figure 1:** PCA Analysis of GSE27515. (a) The normalization of the datasets, and (b) the normalization with respect to the significant gene.

**Figure 2:** Volcano plot.

**Figure 3:** Expression pattern of RAC2 gene.

**Figure 4:** ORA heat-map clustering.

**Figure 5:** ORA pathway enrichment analysis.

**Figure 6:** Biological process of the genes.

**Figure 7:** Cellular component organization.

**Figure 8:** Pathway ontology of genes.

**Figure 9:** ORF Finder.

**Figure 10:** PCR amplification of Rac2 gene. (a) The standardization of the RAC2 that was done using the gradient PCR method. After standardization of the gene, it was compared with the 1 kb DNA ladder. From figure (b), it is clear that the amplified product is above 400 base pairs.

## Data Availability

The data used to support the findings of this study are available from the corresponding author upon request.
